RETRACTED

# Effect of Laparoscopy Combined with Choledochoscope for the Treatment of Cholecystolithiasis and Choledocholithiasis

**DOI:** 10.1155/2022/9110676

**Published:** 2022-06-03

**Authors:** Chengxin Zhang, Qingmei Deng, Jian Zhang, Duofu Li, Bin Fan, Jinman Fang

**Affiliations:** ^1^The First Department of General Surgery, Suzhou First People's Hospital, Anhui Province, Suzhou, Anhui 234000, China; ^2^Hefei Cancer Hospital, Chinese Academy of Sciences, Hefei, Anhui 230000, China; ^3^Institute of Health and Medical Technology, Hefei Institutes of Physical Science, Chinese Academy of Sciences, Hefei, Anhui 230000, China; ^4^University of Science and Technology of China, Hefei, Anhui 230000, China

## Abstract

**Objective:**

Evaluate the influence of laparoscopy combined with choledochoscopy on operation-related indexes, serum total bilirubin (TBIL) level, and abdominal drainage tube extraction time within cases carrying cholecystolithiasis/choledocholithiasis.

**Methods:**

86 cases of cholecystolithiasis together with choledocholithiasis were chosen for this investigation, and cases were randomly segregated within the control cohort (43 cases, open surgery) and observation cohort (43 cases, laparoscopy combined with choledochoscopy).The operation-related indexes, complete stone clearance rate, postoperative visual analogue scale (VAS) scoring, serum TBIL level, and postsurgical complications/recovery incidence were observed and comparatively analyzed across cohorts.

**Results:**

Compared with the control cohort, the incision length, operation duration, postoperative exhaust duration, abdominal drainage tube extraction time, and postsurgery hospitalization in observation cohort were markedly reduced (*P* < 0.05), the intrasurgical hemorrhaging was markedly reduced (*P* < 0.05), and the postoperative complication incidences were markedly reduced (*P* < 0.05). Furthermore, the complete stone clearance rates in the observation cohort were elevated compared with control, but the difference was not statistically significant (*P* > 0.05).VAS scoring for the observation cohort at 6, 12, 24, and 48 hours postsurgery was markedly reduced (*P* < 0.05). On the first day after the operation, the serum TBIL levels for the two cohorts were very high and gradually decreased, and the serum TBIL levels in the observation cohort were markedly reduced during day 1, 3, and 5 postsurgery (*P* < 0.05).

**Conclusion:**

Laparoscopy combined with choledochoscopy surgical treatment might reduce the surgery duration, intrasurgery hemorrhaging, postsurgical pain, and liver function damage.

## 1. Introduction

Cholecystolithiasis is a common clinical disease, and its occurrence is often accompanied by choledocholithiasis, which is characterized by a short course of the disease and apparent abdominal pain symptoms [1]. Recently, with increasing annual incidences of cholecystolithiasis, case quantities with cholecystolithiasis complicated with choledocholithiasis have also increased significantly. If not treated in time, it may induce bile duct edema and pancreatic diseases, affecting everyday lives in typical cases and are life-threatening in severe clinical cases [2]. At present, the most effective treatment for cholecystolithiasis combined with choledocholithiasis is still surgery. However, surgical trauma has a significant inhibiting effect on the immune function of the body, especially open surgery, which often leads to complications such as incision and abdominal infection due to the extensive surgical trauma, seriously affecting the surgical results [3, 4]. Due to emerging advances in surgical techniques, minimally invasive protocols represented by laparoscopy and choledochoscope have gradually been applied to abdominal operations such as cholecystectomy [5]. In this study, by comparing laparoscopic combined choledotoscopy and laparotomy in complete stone clearance, serum TBIL level, and postoperative complications, we probe application influences for laparoscopic/choledotoscopy combinatory procedure within cases carrying cholecystolithiasis complicated with choledocholithiasis. We then provide help for treating cases of cholecystolithiasis aggravated by choledocholithiasis.

RETRACTED

## 2. Material and Methods

### 2.1. Inclusion and Exclusion Criteria

Inclusion criteria are as follows: ① all cases were confirmed to have cholecystolithiasis complicated with choledocholithiasis by imaging examination; ② no contraindications of anesthesia and operation; ③ elective operations; and ④ cases and their families voluntarily participated in study, knew the risks of surgery, and signed the consent form. Exclusion criteria are as follows: ① those who had a history of abdominal surgery such as appendectomy and biliary tract surgery within past; ② those with other biliary tract diseases such as biliary tract polyps and biliary tract strictures; ③ those with incomplete clinical data; ④ those with dysfunction of essential organs such as kidneys and lungs; and ⑤ pregnant or breastfeeding women. This study was approved by our hospital's Medical Ethics Committee.

### 2.2. Research Subjects

According to the above inclusion and exclusion criteria, 86 cases of cholecystolithiasis/choledocholithiasis receiving surgery in our hospital between October 2017 and October 2020 were chosen for this investigation. Among them, there were 39 males and 47 females; the age was 30-70 years, with a mean age of 49.52 ± 13.80 years old; the body mass index (BMI) was 18-27 kg/m^2^, with a mean of 23.05 ± 3.77 kg/m^2^; 30 cases consisted of single gallstone, while 56 patients had several gallstones. Using the random number table method, 86 cases were segregated in significant variations within gender, age, BMI, and gallstones across both cohorts (*P* > 0.05) that were compared (Table 1).

RETRACTED

### 2.3. Surgical Methods

The cases within the control cohort underwent laparotomy. Generalized anesthesia with endotracheal intubation was performed, an oblique incision was made 2 cm below the costal margin for the case's right upper abdomen, and the gallbladder was extracted through laparotomy. Intraoperation, the anterior wall of the common bile duct was cut longitudinally when the stones were found, and the stones within the common bile duct were extracted. After no stone remained within the common bile duct was detected, the “T”-tube was routinely inserted to achieve drainage, the common bile duct was sutured, and the abdomen was closed once the abdominal drain tube was inserted. The observation cohort was treated by laparoscopy combined with choledochoscopy. General anesthesia with endotracheal intubation was performed, a 3-hole protocol was employed for accessing the abdomen, the gallbladder triangle was dissected, and the gallbladder artery and duct were separated. The cystic artery was cut off by an ultrasonic scalpel or electrocoagulation hook, and the cystic duct was clamped and pulled on the anterior wall for the cystic duct to avoid small stones within the gallbladder entering the common bile duct. The choledochoscope was placed within the common bile duct for exploration through the subxiphoid puncture hole, with stones being removed after finding the stones. After successful stone removal, the common bile duct was washed with normal saline through the catheter. At the same time, choledochoscopy was used to check whether there was any residual stone. If there was no residual stone, a “T”-shaped tube was inserted, a common bile duct incision was sutured, and puncture holes within the abdominal wall were closed after placing the abdominal cavity drainage tube. Both cohorts were routinely treated with antibiotics for 3-5 days postsurgery, and “T” tube angiography was performed 1-month postsurgery. “T” tube was removed once the common bile duct was unobstructed, and no stone remained.

### 2.4. Observation Indexes

(1) Operation-related indexes. Incision length, intrasurgical hemorrhage, surgery duration, and postsurgical exhaust duration for two cohorts were observed. (2) Comprehensive stone clearance rate. Stone clearance for cases within two cohorts was analyzed, with the complete stone clearance rate calculated. (3) Postoperative pain. The visual analogue scale (VAS) was employed for evaluating pain for cases at 6, 12, 24, and 48 hours postsurgery, with a maximum individual scoring of 10 points (0 = no pain). (4) Serum TBIL level. The fasting venous blood was extracted from individual cases prior to 1, 3, and 5 days postsurgery, centrifuged at 3000 revs/min (centrifugation radius of 15 cm) for ten minutes, and serum TBIL levels were determined by automatic electrochemiluminescence analyzer. (5) Incidence of postoperative complications. Postoperative complications included incision infection, abdominal infection, biliary bleeding, biliary leakage, and high fever. The incidence of total complications was calculated. (6) Postoperative recovery. The time of abdominal drainage tube removal and postoperative hospital stay were compared across both cohorts

RETRACTED

### 2.5. Statistical Methods

SPSS 22.0 was employed. Count datasets were described by the composition ratio (%)/chi-square test was employed for comparative analyses. Measured datasets fell in line with normal distribution and were reflected through $\bar{x}\pm s$. Comparative analysis across cohorts was performed through *t*-test, the comparison across different time points was performed by one-way ANOVA, and the SNK-q method was employed for pairwise comparison upon the manifestation of variations. *P* < 0.05 was deemed to confer statistical significance.

## 3. Results

### 3.1. Comparison of Surgery-Linked Indexes across Both Case Cohorts

As shown in Table 2, we found the incision length, surgery duration, and postsurgery exhaust duration for the observation cohort were markedly reduced in comparison to the control cohort (*P* < 0.05), and the intrasurgical hemorrhage was markedly reduced in comparison to the control cohort (*P* < 0.05).

### 3.2. Comparison of Complete Stone Clearance Rate across Both Case Cohorts

The complete stone clearance rate for the control cohort was 88.37% (38/43), and that for the observation cohort was 97.67% (42/43). The complete stone clearance rate within the observation cohort was elevated in comparison to the control cohort, though with a nonstatistically significant level of variations (*χ*^2^ = 1.613, *P* = 0.204).

### 3.3. Comparison of Postoperative VAS Scores across Both Case Cohorts

As shown in Table 3, VAS scorings for the observation cohort at 6, 12, 24, and 48 hours postsurgery were markedly reduced in comparison to the control cohort (*P* < 0.05).

### 3.4. Comparison of Serum TBIL Levels before and after Surgery across Both Cohorts

No significant variations were observed for serum TBIL levels across both cohorts prior to surgery (*P* > 0.05). Upon day 1 postsurgery, serum TBIL levels within both cohorts peaked and then slowly reduced, with serum TBIL levels within the observation cohort being significantly lower in comparison to the control cohort during day 1, 3, and day 5 postsurgery (*P* < 0.05) (Table 4).

RETRACTED

### 3.5. Comparative Analysis for Postsurgery Complications

As shown in Table 5, the overall incidence rate for postsurgery complications within the observation cohort was 6.98%, which was markedly reduced compared to the control cohort, which was 23.26% (*P* < 0.05).

### 3.6. Postoperative Recovery across Both Cohorts

As shown in Table 6, we found that the duration for removal of abdominal drain tube/postsurgical hospitalization within the observation cohort was markedly reduced compared to control cohort (*P* < 0.05).

## 4. Discussion

Surgery remains the definitive therapy for cases of cholecystolithiasis complicated with choledocholithiasis. Traditional open cholecystectomy and choledocholithiasis combined with “T” tube drainage can effectively remove stones in cases and reduce postoperative biliary leakage, with clinical effects. However, the trauma of open surgery is relatively significant, and there are disadvantages such as susceptibility to infection, long hospitalization time, and slow recovery [6]. The technology of laparoscopy combined with choledochoscopy is relatively mature, which significantly reduces trauma and relieves pain in cases [7]. Therefore, this study compared the effect of laparoscopy combined with choledochoscopy and open surgery for treating cholecystolithiasis aggravated by choledocholithiasis, aiming to find a less invasive, safe, and effective treatment method for cases.

The application of choledochoscopy within choledocholithiasis can markedly reduce surgery duration and reduce residual bile duct stones and is the leading technology to improve surgical success rates [8]. Application of laparoscopy combined with choledochoscopy can effectively avoid complete dissection and suture for common bile duct, with advantages of minor trauma and complete stone removal [9]. Dataset outcomes from this investigation demonstrated that incision length, operation duration, and postoperative exhaust time of cases treated by laparoscopy combined with choledochoscopy were shorter than open surgery. The intrasurgery hemorrhage was reduced in comparison to open surgery. This result was consistent with the report of Chen et al. [10], which may be related to the minor trauma of this surgical method and the application of choledochoscopy. The dataset outcomes from this investigation revealed that the complete stone clearance rate within the observation cohort was elevated compared to the control cohort. However, such a difference was not statistically significant, suggesting that laparoscopy combined with choledochoscopy and open surgery can effectively remove stones, but the complete stone clearance rate of laparoscopy combined with choledochoscopy was relatively better. Pain is a common postoperative complication, and the pain degree of cases is related to the size of surgical trauma and bile duct injury [11]. Zhang et al. [12] found that VAS scores at 3 and 7 days postcholedochoscopy were markedly reduced compared to cases without choledochoscopy. The dataset outcomes from this investigation revealed that VAS scores of cases with laparoscopy combined with choledochoscopy were lower than those of cases with open surgery at different postoperative time points (6, 12, 24, and 48 hours after operation), like the study of Zhang et al. [12], suggesting that laparoscopy combined with choledochoscopy can significantly reduce postoperative pain in cases with cholecystolithiasis complicated with choledocholithiasis.

RETRACTED

Laparoscopy combined with choledochoscopy and open surgery requires endotracheal intubation for general anesthesia, significantly affecting liver blood circulation and stimulating the body to produce endocrine hormones, resulting in impaired liver function [13]. Guan et al. [14] found that the serum TBIL level in cases treated with laparoscopic cholecystectomy increased significantly on the 1st day after surgery but was lower than that in cases treated with open cholecystectomy and gradually decreased on the seventh day after surgery. However, the decrease was more evident in cases treated with laparoscopic cholecystectomy. Serum TBIL level was used as an indicator to evaluate liver function. This study showed that serum TBIL levels in both cohorts rose to the highest level on the first day after the operation and then gradually decreased. Serum TBIL level in the observation cohort was markedly reduced compared to the control cohort at 1, 3, and 5 days postsurgery, like Guan et al. [14]. Laparoscopy combined with choledochoscopy has sling damage to patient liver function, possibly linked to minor pulling or squeezing of the liver during laparoscopy combined with choledochoscopy [15]. This investigation also identified that the incidence of total postsurgical complications within the observation cohort was markedly reduced compared to the control cohort, similar to Liu et al. [16], suggesting that laparoscopy combined with choledochoscopy within the treatment of cholecystolithiasis and choledocholithiasis is relatively safe. In addition, by comparing the time of removal of abdominal drain tube and postsurgical hospitalization across both cohorts, this study found that the time of removal of abdominal drain tube and postsurgical hospitalizations were shorter within the observation cohort, suggesting that laparoscopic combined with choledochoscopy is beneficial to the postoperative recovery of cases.

RETRACTED

In conclusion, laparoscopy combined with choledochoscopy for treating cases of cholecystolithiasis aggravated by choledocholithiasis has better operation-related indexes than open surgery, with less postoperative pain, less impact on liver function, and high safety, leading to the postsurgery recovery of clinical cases and has specific clinical promotion value.

## Figures and Tables

**Table 1:** Clinical case profile comparative analysis ($n/\left(\bar{x}\pm s\right)$).

Cohort	*n*	Gender		Age (years)	BMI (kg/m^2^)	Gallstones	
		Male	Female			Single	Multiple
Control	43	21	22	49.16 ± 13.39	22.84 ± 4.03	14	29
Observation	43	18	25	50.07 ± 14.25	23.16 ± 3.57	16	27
*t*/*χ*^2^ value		0.422		0.305	0.390	0.205	
*P* value		0.516		0.761	0.698	0.651	

**Table 2:** Comparative analysis for operation-related indexes across both case cohorts ($\bar{x}\pm s$).

Cohort	*n*	Incision length (cm)	Intraoperative blood loss (mL)	Operation time (min)	Postoperative exhaust time (h)
Control cohort	43	11.98 ± 3.74	80.12 ± 23.56	127.30 ± 38.62	44.18 ± 13.50
Observation cohort	43	3.55 ± 1.16	34.91 ± 10.48	86.99 ± 25.01	20.27 ± 6.46
*t* value		14.117	11.497	5.745	10.476
*P* value		0.000	0.000	0.000	0.000

**Table 3:** Comparison of postoperative VAS scores across both case cohorts ($\bar{x}\pm s$, points).

Cohort	*n*	6 hours after operation	12 hours after operation	24 hours after operation	48 hours after operation
Control cohort	43	4.30 ± 1.19	5.57 ± 1.47	5.61 ± 1.52	5.09 ± 1.33
Observation cohort	43	2.56 ± 0.68	3.39 ± 0.90	2.53 ± 0.66	2.28 ± 0.60
*t* value		8.325	8.294	12.188	12.629
*P* value		0.000	0.000	0.000	0.000

**Table 4:** Comparison of serum TBIL levels prior/postsurgery across both cohorts ($\bar{x}\pm s$, *μ*mol/L).

Cohort	*n*	Prior to surgery	Day 1 postop	Day 3 postop	Day 5 postop
Control cohort	43	8.65 ± 2.30	27.01 ± 6.92	20.85 ± 5.31	18.01 ± 4.62
Observation cohort	43	8.97 ± 2.34	23.03 ± 5.87	17.46 ± 4.49	13.79 ± 3.50
*t* value		0.640	2.876	3.197	4.774
*P* value		0.524	0.005	0.002	0.000

**Table 5:** Comparison of postoperative complication rates between the two cohorts (*n* (%)).

Cohort	*n*	Incision infection	Abdominal infection	Biliary tract hemorrhage	Biliary leakage	High fever	Total complication rate
Control cohort	43	3 (6.98)	2 (4.65)	2 (4.65)	1 (2.33)	2 (4.65)	10 (23.26)
Observation cohort	43	0 (0.00)	0 (0.00)	0 (0.00)	2 (4.65)	1 (2.33)	3 (6.98)
*χ* ^2^ value							4.440
*P* value							0.035

RETRACTED

**Table 6:** Postoperative recovery for both case cohorts ($\bar{x}\pm s$).

Cohort	*n*	Time of removal of abdominal drainage tube (d)	Postoperative hospital stay (d)
Control cohort	43	4.08 ± 1.10	10.96 ± 2.81
Observation cohort	43	2.64 ± 0.73	7.12 ± 1.92
*t* value		7.153	7.399
*P* value		0.000	0.000

## Data Availability

The labeled dataset used to support the findings of this study are available from the corresponding author upon request.
